The article "MiR-519b-3p Inhibits the Proliferation and Invasion in Colorectal Cancer via Modulating the uMtCK/Wnt Signaling Pathway" was retracted in 2023. Reasons: original data or images not available; unreliable data; unreliable results or conclusions; concerns about the images.

# MiR-519b-3p Inhibits the Proliferation and Invasion in Colorectal Cancer *via* Modulating the uMtCK/Wnt Signaling Pathway

**DOI:** 10.3389/fphar.2019.00741

**Published:** 2019-07-02

**Authors:** Yuexiang Zhang, Miao Sun, Yusha Chen, Bixun Li

**Affiliations:** ^1^Department of Comprehensive Internal Medicine, Affiliated Tumor Hospital of Guangxi Medical University, Nanning, China; ^2^College of Pharmacy, Guangxi Medical University, Nanning, China

**Keywords:** colorectal cancer (CRC), ubiquitous mitochondrial creatine kinase (uMtCK), proliferation, invasion, carcinogenesis

## Abstract

Dysregulation of microRNAs (miRNAs) and their targeted downstream genes is involved in the carcinogenesis and progression of colorectal cancer (CRC). miR-519b-3p has been reported to play an important role in several cancers. However, its function in CRC is unclear. In this study, we detected the expression of miR-519b-3p in CRC tissues and cell lines, and determined the potential role of miR-519b-3p in cell proliferation and invasion in CRC. Also, the downstream gene of miR-519b-3p was determined. Our results showed that miR-519b-3p was notably reduced in CRC specimens and cell lines. Overexpression of miR-519b-3p inhibited the proliferation and invasion of RKO and DLD-1 cells, whereas knockdown of miR-519b-3p had the contrary effect. The ubiquitous mitochondrial creatine kinase (uMtCK) was identified as a direct target of miR-519b-3p in CRC using luciferase assay. Additionally, miR-519b-3p expression was negatively correlated with uMtCK expression in CRC specimens. Notably, the miR-519b-3p suppressed the uMtCK/Wnt signaling pathway in CRC cells, thereby suppressing CRC cell proliferation and invasion. The inhibition of uMtCK by miR-519b-3p may provide a promising option for the treatment of CRC.

## Introduction

Colorectal cancer (CRC) is one of the most common cancer types globally, with 1.2 million new diagnosed cases as well as 600,000 fatalities annually (Siegel et al., 2015; Moriarity et al., 2016). The morbidity and mortality were reduced in recent years, which probably benefited from the novel effective antitumor drugs and prevention strategies (Kinzler et al., 1991; Zhai et al., 2017). Changes at the molecular level usually occur in CRC and identification of new biomarkers further decreases the morbidity and mortality rates (Ma et al., 2012). The 5-year survival rate of CRC patients has been notably decreased; however, CRC still imposes a huge economic burden on the society (Kong et al., 2018). Therefore, it is urgent to explore new optimal therapeutic strategies to increase the treatment of this disease.

MicroRNAs (miRNAs) are a class of small, single-strand, non-coding RNA with 18–25 nucleotides in length (Asangani et al., 2008). They bind to the three prime untranslated region (3′-UTR) segments of messenger RNAs, inhibiting the expression of target genes in human cancers, including CRC, in which they act as tumor suppressor genes or oncogenes (Liao et al., 2013). Increasing number of studies show that miRNA dysregulation occurs in both early and late stages of CRC. Dysregulation of these miRNAs could induce cell proliferation, apoptosis, angiogenesis, and metastases in CRC (Chen et al., 2009; Tsang and Kwok, 2009). Understanding of the functional mechanism of miRNAs in CRC pathogenesis will be beneficial for the exploration of miRNA-based treatment for CRC.

A recent study has shown that miR-519b-3p, a novel cancer-associated miRNA, also existed in CRC (Luo et al., 2018). However, the function and mechanism of miR-519b-3p in CRC remain unclear. In this study, we investigated the anti-cancer activity of miR-519b-3p in CRC. Our data showed that miR-519b-3p expression was reduced in CRC cell lines and tissues. Overexpression of miR-519b-3p suppressed the invasion and proliferation of CRC cells. Creatine kinases (CKs) are isoenzymes that catalyze the reversible transfer of phosphate groups from phosphocreatine to ADP, generating ATP and creatine (Paltrinieri et al., 2017). Different types of CKs are found in the cytosol and mitochondria of cells. There are two types of mitochondrial CKs (MtCKs), sarcomeric MtCK (sMtCK) and ubiquitous MTCK (uMtCK), which are encoded by two genes and expressed in a tissue-specific manner (Hoshino et al., 2009). uMtCK has been shown to be involved in several cancers, such as prostate cancer, hepatocellular carcinoma, and breast cancer (Qian et al., 2012; Uranbileg et al., 2014; Amamoto et al., 2016). Interestingly, we identified UMTCK as a target gene of miR-519b-3p in CRC. Moreover, we found that overexpression of miR-519b-3p negatively regulated Wnt signaling in CRC cells. Our findings illustrated that miR-519b-3p impeded cell invasion and proliferation in CRC *via* targeting UMTCK/Wnt signaling, which might be considered as a potential target for CRC therapy.

## Materials and Methods

### Tissue Specimens

A total of 48 CRC tissues and paired surrounding non-tumor tissues were harvested from patients undergoing surgical resection at the Affiliated Tumor Hospital of Guangxi Medical University during May 2016 to December 2017. Isolated tissues were immediately transferred into and stored in liquid nitrogen at −80°C. All subjects signed informed consent forms and agreed. Our study was approved by the Human Trial Ethics Committee of the Affiliated Tumor Hospital of Guangxi Medical University. All experiments were conducted in accordance with the Declaration of Helsinki.

### RNA Extraction and qRT-PCR

Total RNA was isolated using TRIzol reagent (Invitrogen, Grand Island, NY). Complete reverse transcription was performed with Transcriptase superscript III (Invitrogen, Grand Island, NY). Quantitative reverse transcriptase PCR (qRT-PCR) was completed with the Bio-Rad CFX96 system, and gene expression levels were detected by SYBR green. qRT-PCR primer sequences were as follows: miR-519b-3p, F, 5′-GGTCAAGTGACACCGTCG-3′, R, 5′-TGCAGCTGGGGGTCAG-3′; uMtCK, F, 5′-TCGTCTGACGGACAAGCG-3′, R, 5′-GGCCGTAGGGGTGATC-3′;GAPDH, F, 5′-CAGCCATTGTACGTCACCCA-3′, R, 5′-GAGTCCTGCGGGTAGG-3′. PCR conditions were as follows: 55°C for 3 min, 95°C for 8 min, and then followed by 95°C for 15 s and 60°C for 15 min, which were performed for 45 cycles. Glyceraldehyde 3-phosphate dehydrogenase (GAPDH) served as an internal reference to analyze the gene expression levels. The experiments were performed in triplicate for each condition.

### Western Blot Analysis

Proteins were split from the splitting buffer and transferred to polyvinylidene fluoride or polyvinylidene difluoride membranes by electrophoresis (Millipore, Billerica, MA). The membrane was blocked with bovine serum albumin (Sigma-Aldrich, St. Louis, MO). Then, the membrane was incubated with primary antibodies at 4°C overnight, followed by incubation with secondary antibodies at room temperature for 60 min. The main antibodies include cleaved uMtCK (Abcam, dilution ratio is 1:1,000) and anti-GAPDH (Abcam, dilution ratio is 1:2,000). Secondary antibodies were rabbit anti-mouse IgG (Abcam, dilution ratio is 1:1,000). Protein bands were visualized by the ECL Chemiluminescence Detection System (Thermo Fisher Science, Rochester, NY). The experiments were repeated three times.

### Cell Counting Kit-8 (CCK-8) Test

Cells (1 × 10^4^ cells/well) were plated and cultured overnight. MiR-519b-3p mimics or inhibitors were transfected to cells. After 48 h, 10 μl of CCK-8 reagent (Sigma, St. Louis, MO, USA) was supplemented. The absorbance was measured at 450 nm (OD) with a microplate reader (BioTek Instruments Inc., Winooski, VT, USA).

### Colony Formation Assay

Cells were transfected with miR-519b-3p mimics or inhibitor. After 48 h, transfected cells were incubated in Dulbecco’s Modified Eagle’s medium substrate with 0.3% soft agar and 10% fetal bovine serum (FBS). Then, cells (1 × 10^3^ cells/well) were plated into 6-well plates, in which DMEM substrate with 10% FBS was supplemented. Two weeks later, the colonies were stained with 0.1% crystal violet dye (Sigma). The mean number of colonies was presented as histograms.

### Transwell Assay

Cells (1 × 10^4^) in serum-free medium were seeded in the upper chamber coated with Matrigel (BD, San Jose, CA, USA) in 24-well plates. The lower chamber was filled with 500 μl of DMEM medium supplemented with 10% FBS. Twenty-four hours later, cells the migrated to the bottom of the chamber were fixed by methanol and stained with crystal violet dye (Sigma). The number of migrated cells was counted under a light microscope.

### Dual-Luciferase Assay

The 3′-UTR fragments of uMtCK cDNA that contained the predicted binding site of miR-519b-3p were cloned into the pmirGLO vector (Promega Biotech Co., Madison, WI, USA). The site-directed mutagenesis of miR-519b-3p binding site on the 3′-UTR of uMtCK was conducted with the Site-Directed Mutagenesis Kit (Stratagene, San Diego, CA, USA). Constructed vectors were co-transfected with miR-519b-3p mimics or inhibitor with Lipofectamine 2000 (Invitrogen) for 48 h. Cells were co-transfected with miR-519b-3p mimics or inhibitor, TOPFlash luciferase reporter, and phRL-TK renilla luciferase reporter (Promega) to detect Wnt signaling activity. Forty-eight hours later, the luciferase activity post-transfection was assessed with the Dual-Luciferase Reporter Assay System (Promega) in compliance with the manufacturer’s instructions.

### Statistical Analysis

Statistical analysis was performed with SPSS version 18.0 (SPSS Inc., Chicago, IL, USA), and the data are shown as mean ± standard deviation. The statistical significance between two groups was analyzed *via t* test. Statistical significance of various groups was analyzed by one-way analysis of variance followed by Bonferroni’s multiple comparison test. Correlation coefficient analysis was performed by Spearman’s rank-order correlation. *p* value < 0.05 was deemed as statistically significant.

## Results

### Down-Regulated Expression of miR-519b-3p in CRC Cell Lines and Tissues

To investigate the effect of miR-519b-3p in CRC, real-time fluorescence-based quantitative PCR was applied to measure the miR-519b-3p expression in CRC tissues. Data illustrated that relative to surrounding non-tumor tissues, miR-519b-3p expression was notably decreased in CRC tissues (**Figure 1A**, *p* < 0.001). Moreover, miR-519b-3p expression in CRC cell lines was also examined. The level of miR-519b-3p in CRC cells was lower than that in normal colonic mucosa epithelial cells (**Figure 1B**). Together, these results suggest that miR-519b-3p expression is down-regulated in CRC, indicating an anti-tumor function of miR-519b-3p in CRC.

**Figure 1:** miR-519b-3p expression was down-regulated in colorectal cancer (CRC). **(A)** Relative expression of miR-519b-3p in CRC tissues and surrounding non-cancerous tissues were detected by qRT-PCR. **p < 0.01 vs. Adjacent. **(B)** Relative expression of miR-519b-3p in CRC cell lines (HT29, RKO, DLD-1, and SW620) and normal colon mucosal epithelial cells NCM460 was measured by qRT-PCR. **p < 0.01, ***p < 0.001 vs. NCM460.

### miR-519b-3p Suppresses the Proliferation and Invasion of CRC Cells

To study the potential anti-tumor effect of miR-519b-3p in CRC, we conducted transient transfection in RKO and DLD-1 cells with miR-519b-3p mimics or inhibitor, followed by the gain-of-function and loss-of-function experiments. Real-time fluorescence-based quantitative PCR showed that miR-519b-3p expression was significantly increased in the miR-519b-3p mimic group (**Figure 2A**). CCK-8 assay showed that miR-519b-3p overexpression suppressed CRC cell proliferation (**Figure 2B**). The colony formation efficiency of CRC cells was also significantly reduced by the overexpression of miR-519b-3p (**Figure 2C**). The inhibitory effect of miR-519b-3p on the invasive capability of cancer cells was measured with Transwell assay. CRC cell invasive ability was significantly inhibited by the overexpression of miR-519b-3p, while the miR-519b-3p inhibitor group showed the opposite effect (**Figure 2D**). These results indicated that in CRC cells, miR-519b-3p possessed potent anti-tumor effect by suppressing cell proliferation and invasion.

**Figure 2:** Overexpression of miR-519b-3p suppressed the proliferation and invasion of CRC cells. **(A)** Expression of miR-519b-3p in RKO and DLD-1 cells transfected with miR-519b-3p mimics or inhibitor was detected by qRT-PCR. **(B)** Cell proliferation was detected in RKO and DLD-1 cells transfected with miR-519b-3p mimics or inhibitor by cell counting kit-8 (CCK-8) assay. **(C)** The colony number was examined in RKO and DLD-1 cells. **(D)** The effect of miR-519b-3p on invasion was examined by Transwell assay. *p < 0.05, **p < 0.01, ***p < 0.001 vs. NC. NC, negative control.

### uMtCK is the Direct Target Gene of miR-519b-3p

To explore the potential anti-tumor mechanism of miR-519b-3p, we performed bioinformatic prediction analysis to predict potential targets of miR-519b-3p using online databases, including microRNA target prediction (http://mirdb.org/) and microRNA.org (http://www.microrna.org/microrna/home.do). Among these targets, uMtCK, which had a high score and has been reported to function in several cancers, was considered to be a potential target of miR-519b-3p in CRC. The 3′-UTR of uMtCK contained a putative binding site of miR-519b-3p (**Figure 3A**). Through the dual-luciferase reporter assay, we investigated whether uMtCK was a direct target gene of miR-519b-3p in CRC. The 3′-UTR fragment of uMtCK, which contains a putative binding site of miR-519b-3p, was cloned into pmirGLO reporter vector. The dual-luciferase assay showed that the luciferase activity was notably decreased with overexpression of miR-519b-3p and elevated with miR-519b-3p inhibition (**Figure 3B and C**). Nevertheless, the activity of mutant luciferase reporters was not impacted by either overexpression or inhibition of miR-519b-3p. Additionally, miR-519b-3p overexpression down-regulated the protein and messenger RNA levels of uMtCK, whereas inhibition of miR-519b-3p increased uMtCK expression at both the protein and mRNA level (**Figure 4A and B**). We also found that the mRNA expression of uMtCK was remarkably up-regulated in CRC tissues (**Figure 5A**). The correlation analysis indicated that the mRNA level of uMtCK was inversely related to the expression of miR-519b-3p (*r* = −0.846, *p* < 0.001, **Figure 5B**). Taken together, our data suggest that uMtCK is a direct target gene of miR-519b-3p.

**Figure 3:** miR-519b-3p could directly target the 3′-UTR of uMtCK. **(A)** The putative miR-519b-3p binding site in the 3′-UTR of uMtCK mRNA. The dual-luciferase reporter assay was used in RKO **(B)** and DLD-1 **(C)** cells transfected with miR-519b-3p mimics or inhibitor. *p < 0.05, **p < 0.01 vs. NC. NC, negative control.

**Figure 4:** miR-519b-3p repressed the expression of uMtCK. Relative mRNA expression levels of uMtCK in RKO and DLD-1 cells transfected with miR-519b-3p were assessed by qRT-PCR. **(B)** Relative protein expression levels of uMtCK in RKO and DLD-1 cells were examined by Western blot. *p < 0.05, **p < 0.01 vs. NC. NC, negative control.

**Figure 5:** uMtCK was negatively correlated with miR-519b-3p expression in CRC tissues. **(A)** Relative mRNA expression of uMtCK in CRC tissues and surrounding non-cancerous tissues was detected by qRT-PCR. ***p < 0.001 vs. Adjacent. **(B)** Correlation between uMtCK mRNA and miR-519b-3p expression was detected by Spearman’s correlation assay. *r* = −0.846; ***p < 0.001.

### miR-519b-3p Abrogates Wnt Signaling *via* uMtCK in CRC Cells

Wnt signaling plays an important role in CRC. Next, we explored the impact of miR-519b-3p on Wnt signaling pathway CRC cells. qRT-PCR results denoted that overexpression of miR-519b-3p down-regulated Wnt signaling pathway (**Figure 6A**). Also, miR-519b-3p overexpression significantly impeded c-myc transcription (**Figure 6B**), as well as cyclin D1 (**Figure 6C**). Together, inhibition of miR-519b-3p dramatically activated Wnt signaling. These findings suggest that miR-519b-3p could modulate the Wnt signaling pathway.

**Figure 6:** miR-519b-3p suppressed Wnt signaling in RKO and DLD-1 cells. **(A)** Relative luciferase activity of Wnt signaling was detected by the Dual-Glo luciferase system. **(B, C)** Relative mRNA expressions of c-myc and cyclin D1 were assessed by qRT-PCR. *p < 0.05 vs. NC. NC, negative control.

### The Recovery of uMtCK Expression Reversed the Anti-Tumor Impact of miR-519b-3p

To confirm whether miR-519b-3p inhibited the proliferation and invasion of CRC cells *via* targeting UMTCK, we transfected CRC cells with pcDNA3.1/UMTCK vector to recover the UMTCK expression in miR-519b-3p mimics-transfected cells. Our findings illustrated that the protein expression levels of uMtCK were dramatically increased in miR-519b-3p mimics-transfected cells after the transfection of pcDNA3.1/UMTCK vector. The recovery of the expression of UMTCK reversed the suppressive effect of miR-519b-3p on Wnt signaling pathway to a large extent (**Figure 7B**). In addition, the recovery of the expression of uMtCK dramatically reduced the suppressive effect of miR-519b-3p on CRC cell proliferation (**Figure 7C**) and invasion (**Figure 7D**). These results indicated that miR-519b-3p inhibits the proliferation and invasion of CRC cells by down-regulation of uMtCK.

**Figure 7:** Restoration of uMtCK expression abolishes the antineoplastic activity of miR-519b-3p. DLD-1 and RKO cells were transfected with miR-519b-3p mimics and pcDNA3.1/uMtCK expression vector and cultured for 48 h. **(A)** Protein expression of uMtCK was detected by Western blot. **(B)** Wnt signaling was examined by TOPFlash reporter assay. **(C)** Cell proliferation was detected by CCK-8 assay. **(D)** DLD-1 and RKO cell invasions were assessed by Transwell invasion assay. *p < 0.05.

## Discussion

Our study confirmed the anti-tumor effect of miR-519b-3p in CRC. Our data showed that miR-519b-3p was dramatically down-regulated in CRC cell lines and tissues, and overexpression of miR-519b-3p suppressed CRC cell proliferation and invasion. Interestingly, we found that uMtCK is a promising new target gene of miR-519b-3p. Overexpression of uMtCK attenuated Wnt signaling activity, and recovery of uMtCK expression inhibited the anti-tumor effect of miR-519b-3p. We demonstrated that miR-519b-3p could serve as an inhibitor of the development of CRC by down-regulating uMtCK.

Due to the heterogeneity of CRC tumor samples, it is quite urgent to identify effective biomarkers. For instance, miR-17-5p, miR-21, miR-224, and miR-429 were up-regulated in CRC, whereas miR-126, miR-330, miR-18-3p, miR-185, miR-320a, miR-143, and were down-regulated (Moridikia et al., 2018). So far, the function of miR-519b-3P is not clear. One study showed that miR-519b-3p, as a novel CRC-related miRNA, could directly bind to ARID4B 3′-UTR mRNA, which was negatively regulated by miR-519b-3p expression (Hoshino et al., 2009). Our study detected decreased miR-519b-3p expression in both CRC cell lines and tissues, and it was consistent with a recent study showing that miR-519 was significantly down-regulated in CRC (Deng et al., 2016). Furthermore, we explored the biological activity of miR-519b-3p in CRC and observed that miR-519b-3p inhibited CRC cell proliferation and invasion. Our data indicated the anti-tumor effect of miR-519b-3p in CRC.

uMtCK has become a new therapeutic target for cancers. In hepatocellular carcinoma cells, uMtCK regulates the key processes of transcription involved in cell proliferation and invasion (Uranbileg et al., 2014). uMtCK is highly expressed in breast cancer cells, while knockdown of uMtCK inhibits cell growth and proliferation (Qian et al., 2012). Pang et al. have shown that stable transfection with exogenous uMtCK promotes tumor growth of LNCaP cells (Pang et al., 2009). We found in this study that uMtCK was the direct target gene of miR-519b-3p in CRC. miRNA usually binds to the 3′-UTR of target mRNAs and causes translation repression or mRNA degradation (Iorio et al., 2005). In this study, we found that miR-519b-3p bound to the 3′-UTR of uMtCK. Moreover, the expression of uMtCK was regulated by miR-519b-3p. These results indicate that miR-519b-3p is a novel upstream regulator of uMtCK. We also observed that the expression of miR-519b-3p was negatively correlated with the level of uMtCK in CRC tissue samples. The reduced expression of miR-519b-3p might induce uMtCK-mediated development of CRC. Thus, inhibiting uMtCK *via* miR-519b-3p may serve as an optimal treatment option for CRC.

The Wnt pathway is a classical signaling pathway in the development of a variety of cancers, with the aberrant activation of Wnt signaling found in nearly 80% of CRC (Mantovani et al., 2018). The activation of adenomatous polyposis coli (APC) gene mutation and β-catenin expression resulted in the aberrant activation of Wnt signaling (Hashimoto et al., 2017). Nevertheless, other mediators such as Wnt ligands and inhibitors were also related to the start of CRC (Hashimoto et al., 2017). We confirmed in our study that miR-519b-3p dramatically deactivated Wnt signaling *via* inhibiting uMtCK, indicating a new alternative pathway regulating Wnt signaling.

To sum up, our study initially confirms that miR-519b-3p is a new anti-cancer miRNA in CRC, which inhibits CRC proliferation and invasion *via* targeting uMtCK. Our findings give insights into the effect of miR-519b-3p/uMtCK in CRC development. miR-519b-3p/uMtCK might act as promising targets in the treatment of CRC.

## Data Availability Statement

The raw data supporting the conclusions of this manuscript will be made available by the authors, without undue reservation, to any qualified researcher.

## Author Contributions

YZ carried out further experiments for manuscript revision, and also revised the manuscript significantly. MS carried out the *in vitro* and *in vivo* studies and drafted the manuscript. YC carried out the luciferase report assay. YC and MS participated in the design of the study and performed the statistical analysis. BL conceived of the study, and participated in its design and coordination and helped to draft the manuscript. All authors read and approved the final manuscript.

## Funding

This study was funded by the Foundation of Guangxi Science and Technology Development Program (no. 1598012-8).

## Conflict of Interest Statement

The authors declare that the research was conducted in the absence of any commercial or financial relationships that could be construed as a potential conflict of interest.
